# The Antisenescence Effect of Exosomes from Human Adipose-Derived Stem Cells on Skin Fibroblasts

**DOI:** 10.1155/2022/1034316

**Published:** 2022-06-29

**Authors:** Ji-An Guo, Pi-Jun Yu, Dong-Qin Yang, Wei Chen

**Affiliations:** ^1^Department of Aesthetic Plastic Surgery, Shanghai Eighth People's Hospital, Shanghai 200235, China; ^2^Department of Hematology, Shanghai Eighth People's Hospital, Shanghai 200235, China

## Abstract

Human adipose-derived stem cells (ADSCs) have become a promising therapeutic approach against skin aging. Recent studies confirm that exosomes partially mediate the therapeutic effect of stem cells. This study successfully isolated exosomes from the ADSC culture medium and discovered that ADSC-derived exosomes (ADSC-Exos) could alleviate human dermal fibroblast (HDF) senescence and stimulate HDF migration. Moreover, ADSC-Exos increased the type I collagen expression level and reduced the reactive oxygen species (ROS) and senescence-associated *β*-galactosidase (SA-*β*-Gal) activity in HDFs. In addition, we demonstrated that ADSC-Exos significantly inhibited senescence-related protein expression levels of p53, p21, and p16. In conclusion, our results have revealed the antisenescence effects of ADSC-Exos on HDFs and ADSC-Exos may be a novel cell-free therapeutic tool for antiaging.

## 1. Introduction

The skin is the barrier between the body and the environment. In addition to protecting the body from water loss and microbial infection, it also has critical cosmetic functions. However, with the increase of age, the skin will also show apparent signs of aging. A series of pathophysiological changes occur in the skin with aging. Wrinkles characterize skin aging, including a decreased volume, loss of elasticity, sagging, and a rough appearance [1]. The skin's ability to heal itself decreases as a person ages. There are many internal and external causes of skin aging [2]. Intrinsic changes are determined by genes, of which posttranslational mechanisms and epigenetic changes are important; on the other hand, extrinsic aging is caused by external factors such as smoking, UV exposure, pollution, and nutritional imbalance [3].

Skin aging is mainly due to the senescence of dermal fibroblasts. As people age, dermal fibroblasts lose their ability to proliferate and synthesize collagen, mainly types I and III, the essential extracellular matrix component of the dermis [4]. Type I collagen, which is involved in skin elasticity, flexibility, and tension, makes up 80% of the total collagen [5]. With age, the activity and number of skin fibroblasts decrease, the formation and repair of the matrix slow down, and the degradation of the existing skin matrix accelerates, ultimately reducing the skin's ability to regenerate [6, 7].

Adipose-derived stem cells (ADSCs), one of the mesenchymal stem cells (MSCs), are among the most widely studied stem cells in recent years [8, 9]. ADSCs possess self-renewal, multiple differentiation potential, and immunomodulatory effects, with favorable functions, such as wound repair, antiaging and antiapoptotic effects via differentiation, or paracrine effect [2–4]. Previous studies have reported that ADSCs can improve photoaging wrinkles and promote collagen production in photoaged fibroblasts in vitro [5, 6]. Despite the tremendous achievements of stem cell therapy, there are still some challenges in clinical application, especially the low survival rate after transplantation [10, 11]. So, there is an urgent need to find better ways to use stem cells in the clinic. Promisingly, accumulating experimental and clinical studies reveal that the paracrine effect, particularly by exosomes, of transplanted stem cells plays a critical role in the therapeutic effect and the change of damaged tissues [10, 12–14].

Recent studies have shown that exosomes derived from MSCs can significantly regulate molecular transport between cells, which may be an essential mechanism for stem cells to play a regulatory role [15, 16]. Exosomes are 30–150 nm extracellular vesicles formed through the process of endocytosis-fusion-effluence of cells and are highly rich in bioactive substances such as nucleic acids, proteins, cytokines, and other molecules [17–19]. Exosomes transport these bioactive factors that target specific recipient cells, trigger downstream signals, or participate in cell-to-cell communication [20]. MSC-derived exosomes (MSC-Exos) have been proposed as a new cell-free treatment for skin regeneration [21]. Therefore, more and more attention has been paid to the clinical application of exosomes [22]. Exosomes can potentially be used for prognosis, therapy, and biomarkers for health and disease [23]. By transferring bioactive substances to fibroblasts, bone marrow MSC-Exos can promote cell migration, proliferation, collagen synthesis, and skin repair and healing [24]. These studies have shown that exosome paracrine from stem cells is essential for the regeneration of tissues or cells. Compared with MSCs, exosomes offer higher therapeutic efficiency and are also more convenient to prepare, store, transport, and administer [25, 26]. In addition, they avoid the risk of immune rejection and tumor development associated with stem cell transplants [27–29]. Therefore, ADSC-derived exosome- (ADSC-Exos-) mediated therapy may be safer and more efficient than ADSC-based therapy. However, the effect of MSC-Exos on skin aging has not been clearly studied.

In this study, we compared the changes in cellular activity and cellular morphology to research the antisenescence effects of ADSC-Exos on skin fibroblasts in vitro. We also investigated aging markers at the protein level and changes in the pathway. Our findings may provide some experimental and theoretical bases for the application of ADSC-Exos in clinical antiaging.

## 2. Materials and Methods

### 2.1. Ethics Statement

This study was performed with permission from the institutional ethics committee of Shanghai Eighth People's Hospital (2020-YS-041). The signed informed consent was received from all patients for the use of their tissues. All the data concerning the donors were anonymized upon collection of surgical residues by surgeons before culturing.

### 2.2. Isolation and Cultivation of ADSCs

Human abdominal fat tissues were obtained from the waste material of three female patients (average age 25 ± 5 years) who underwent liposuction. The subcutaneous fat was washed three times with phosphate-buffered saline (PBS) (HyClone, Logan, UT, USA) containing 100 U/mL penicillin and 100 *μ*g/mL streptomycin (Gibco, Grand Island, NY, USA) and gently shaken to remove blood. Adipose tissues were then treated with 0.1% type I collagenase (Sigma-Aldrich, St. Louis, MO, USA) and incubated for 40 minutes at 37°C in a constant temperature oscillation incubator. Then, Dulbecco's modified Eagle medium/nutrient mixture F12 (DMEM/F12; Gibco) containing 10% fetal bovine serum (FBS) (Gibco), 100 U/mL penicillin, and 100 *μ*g/mL streptomycin was added to stop the digestion. The digested fat was centrifuged at 300 × g for 10 minutes. The supernatant was discarded, and the pellet was resuspended in the complete medium (DMEM/F12 containing 10% FBS) and filtered through a 100 *μ*m nylon mesh filter (Millipore, Billerica, MA, USA). The filtered cell fraction was incubated overnight, and the adherent cells were collected, maintained in an incubator at 37°C in a humidified atmosphere containing 5% CO_2_, and cultured to passage 3 for experiments.

### 2.3. Immunophenotype Characterization of ADSCs

To characterize the ADSCs, we performed a flow cytometric analysis for four MSC markers, CD44, CD73, CD90, and CD105, and two negative markers, CD34 and CD45. Fluorescence-conjugated antibodies were purchased from eBioscience (San Diego, CA, USA). The surface antigens were analyzed with a FACSVerse system (BD Bioscience, San Jose, CA, USA) using FlowJo software (TreeStar Inc., San Carlos, CA, USA).

### 2.4. Adipogenic and Osteogenic Differentiation and Authentication of ADSCs

ADSCs in passage three were subjected to stem cell induction and appraisal system to examine ADSCs' differentiation ability. For adipogenic differentiation ability, ADSCs were seeded at 2 × 10^4^ cells/cm^2^ in 6-well cell culture plates. Cells were allowed to grow to post confluence in the complete medium. Adipogenic differentiation of ADSCs was achieved using an adipogenic kit (Cyagen Biosciences, Guangzhou, China) and was confirmed by oil red O (Cyagen) staining of lipid droplets after 16 days in culture.

For osteogenic differentiation of ADSCs, cells were seeded at 2 × 10^4^ cells/cm^2^ in 6-well cell culture plates precoated with 0.1% gelatin solution (Cyagen). Cells were grown to 80%–90% confluence in the complete medium and then replaced with osteoinduction medium (Cyagen). Osteoinduction was stopped on day 18, and the cells were stained with alizarin red (Cyagen) for microscopic visualization.

### 2.5. Isolation of ADSC-Exos

Exosomes were isolated from the medium of ADSCs as previously described [30]. ADSCs were cultured in serum-free DMEM/F12 for 24 h to collect the medium. The medium was centrifuged at 300 × g for 10 min and 2000 × g for 10 min to eliminate dead cells and cell debris. Then, the supernatant was centrifuged at 10000 × g for 30 min and 110000 × g for 70 min to collect exosomes in an ultracentrifuge (Beckman L-100, Beckman Coulter, Brea, CA, USA). The pellets were resuspended in 2 mL PBS and reultracentrifuged at 110000 × g for 70 min. The pelleted exosomes were resuspended in PBS and stored at −80°C or used for subsequent experiments. All procedures were conducted at 4°C.

### 2.6. Identification of ADSC-Exos

The morphological analysis of ADSC-Exos was conducted using the transmission electron microscope (TEM) (Hitachi, Tokyo, Japan). The size distribution and concentration of ADSC-Exos were measured by nanoparticle tracking analysis (NTA) using the NanoSight system (NanoSight; Wiltshire, UK). ADSC-Exos were diluted with PBS (1 : 1000) and mixed well into individual pellets. Carefully inject the diluted exosomes into the NanoSight instrument using a syringe, avoiding the generation of microscopic air bubbles. The Brownian motion of each nanoparticle of exosomes can be observed using NanoSight, and the concentration and size distribution of exosomes can be calculated by NTA. Exosome marker proteins CD9, CD63, and CD81 (Abcam, Cambridge, UK) were analyzed by Western blot analysis (these methods were described in more detail as follows).

### 2.7. Isolation and Cultivation of HDFs

Dermal fibroblasts were obtained from the skin of three elderly (aged >60 years) healthy women undergoing breast reduction plastic surgery. Briefly, fibroblasts migrated from 1 mm diameter biopsies taken from the skin samples and were cultured in Dulbecco's modified Eagle's medium (DMEM) (Gibco) supplemented with 10% FBS, 100 U/mL penicillin, and 100 *μ*g/mL streptomycin in a 90% humidified incubator with 5% CO_2_ at 37°C. Cells were amplified, weekly passaged at 80%–90% confluence, and used at early (between the 2nd and the 4th) passages to avoid in vitro replicative-induced senescence. Passage three HDFs were used in all experiments and were seeded at a density of 5 × 10^4^ cells/cm^2^ unless otherwise stated.

### 2.8. Cell Proliferation Assay

Cell proliferation was determined using a Cell Counting Kit-8 assay (CCK-8) (Dojindo Laboratories, Kumamoto, Japan) following the manufacturer's instructions. HDFs were allocated into ADSC-Exos or PBS groups. Each group of cells had three replicates seeded in 96-well plates (5 × 10^3^ cells/well). Add 100 *μ*L of DMEM with 10% FBS to each well and incubate overnight to allow cells to adhere. Subsequently, cells in the ADSC-Exos group were treated with the final concentration of 20 *μ*g/mL ADSC-Exos for 0, 24, 48, and 72 h. The PBS group was treated with PBS for 0, 24, 48, and 72 h. CCK-8 solution was then added to each well and incubated for 2 h at 37°C. The optical density (OD) at 450 nm was measured using a microplate reader (S/N 415-2687, Omega Bio-Tek, Ortenberg, Germany).

### 2.9. Cell Migration Assays

Plate the HDFs in 12-well plates and incubate at 37°C. After cells attach, scrape the confluent monolayer using a 200 *μ*L pipette tip and wash with PBS to remove cellular debris and smooth the edges of the scratch. 2 mL of serum-free DMEM media containing exosomes or PBS was added. Cells were photographed immediately (*t* = 0 h), 12 hours (*t* = 12 h) and 24 hours (*t* = 24 h) later. The level of the migration area was assessed by the ratio of the closure area to initial wound (*t* = 0 h) as follows: migration area (%) = (*A*0 − An)/*A*0 × 100, where *A*0 represents the area of the initial wound area and An represents the residual area of the wound at the metering point (*t* = *n* h).

### 2.10. Reactive Oxygen Species (ROS) Content Assay

The intracellular ROS levels were analyzed by the ROS assay kit (Beyotime, Shanghai, China), as Liao et al.'s article described [31]. HDFs were seeded at a 1 × 10^5^/well density in 35 mm diameter confocal dishes and incubated for 24 hours. Afterward, 25 mM 2′-7′-dichlorofluorescein diacetate (DCFH-DA) was added and the cells were incubated at 37°C for 30 min. The ROS content of HDF was then observed by an LSM780 confocal microscope (Zeiss, Germany) at 488 nm excitation and 525 nm emission wavelength.

### 2.11. Senescence-Associated *β*-Galactosidase (SA-*β*-Gal) Staining

SA-*β*-Gal staining was used to determine the effects of ADSC-Exos on the cell senescence of HDFs. ADSC-Exos-treated HDFs were seeded at a 5 × 10^4^/well density in 6-well plates with the culture medium and incubated at 37°C and 5% CO_2_ for 24 hours. Afterwards, the cells were fixed with 4% paraformaldehyde (PFA) (Sigma-Aldrich) at room temperature for 20 min and subsequently stained by the SA-*β*-Gal staining kit (Beyotime) following the manufacturer's instructions. Positive senescent cells stained in blue were observed using an inverted microscope (Zeiss), as described in the previous researcher's writing [31]. Three images per well were collected, and the SA-*β*-Gal-stained cells were counted. The corresponding quantification of the SA-*β*-Gal staining was analyzed by ImageJ (National Institutes of Health).

### 2.12. Type I Collagen ELISAs

The effect of ADSC-Exos on the collagen synthesis capacity of HDFs was detected by enzyme-linked immunosorbent assay (ELISA). First, seed HDFs in 6-well plates and add 2.5 mL of DMEM containing 10% FBS to each well. After HDFs were cultured for 72 hours or reached 80% confluence, ADSC-Exos or PBS were added for coculture for 72 hours. Afterward, the conditioned medium was collected and collagen type I levels were quantified using an ELISA kit (Abcam). Measure the absorbance at 450 nm using a microplate reader (S/N 415–2687).

### 2.13. Western Blot Analysis

Add RIPA buffer (CST, USA) containing protease inhibitors to the three groups of HDFs and use an ultrasonic cell disruptor to lyse the cells fully. The lysate was centrifuged, and the pellet was discarded. The protein sample concentration was detected using a BCA protein assay kit (Beyotime). Equal amounts of protein were electrophoretically separated using a preprepared 12% SDS-polyacrylamide gel (SDS-PAGE). After electrophoresis, proteins were transferred to polyvinylidene fluoride (PVDF) membranes (Millipore, USA) and incubated with corresponding primary and secondary antibodies. Target bands of proteins were scanned using an ImageQuant LAS 4000 Chemiluminescence Imager (GE, USA). Primary antibodies to CD9, CD63, and CD81 were purchased from Abcam, and primary antibodies to human p16, p21, p53, and *β*-actin and all secondary antibodies were purchased from Beyotime.

### 2.14. Statistical Analysis

Statistical analysis was performed using the Statistical Program for Social Science (SPSS) software 20.0 package (SPSS, Chicago, IL, USA). All results are expressed as the mean ± SD of at least 3 independent experiments and were compared with two-tailed Student's *t*-tests. *P* values < 0.05 were considered statistically significant.

## 3. Results

### 3.1. Identification of ADSCs

The ADSCs were characterized morphologically by a small cell body with a few cell processes that were long and thin. The cell body contains a large, round nucleus with a prominent nucleolus, surrounded by finely dispersed chromatin particles, giving the nucleus a clear appearance (Figure 1(a)). Flow cytometry was used to evaluate the expression of cell surface antigens for ADSCs at passage 3. The results showed that the ADSCs expressed CD44, CD73, CD90, and CD105 with minimal expression of CD34 and CD45 (Figure 1(b)). To identify the multipotency of ADSCs, adipogenic differentiation and osteogenic differentiation of these cells were assessed using oil red O and alizarin red staining (Figures 1(c) and 1(d)) and we authenticated the accumulation of lipid vacuoles in differentiated adipocytes and calcium precipitation of osteocytes, respectively. Therefore, these data indicate that ADSCs have been successfully isolated.

### 3.2. Identification of ADSC-Exos

Exosomes were isolated from the ADSCs by ultracentrifugation. The isolated ADSC-Exos were verified as small vesicles of approximately 100 nm in size using the transmission electron microscopy (TEM) assay (Figure 2(a)). The size distribution and concentration were analyzed using nanoparticle tracking analysis (NTA). The isolated ADSC-Exos had a predominant size of 95.16 nm, which was in accord with the feature of exosome (30–150 nm) and a concentration averaging around 1.73 × 10^8^/mL (Figure 2(b)). Exosome surface markers CD9, CD63, and CD81 also presented higher expression than ADSCs (Figure 2(c)).

### 3.3. Proliferation and Migration of Senescence HDFs Were Promoted by ADSC-Exos

After 0, 24, 48, and 72 hours of coculture with ADSC-Exos or PBS (control), the proliferative capacity of the three groups of senescence HDFs was determined by the CCK-8 assay. The results indicated that the proliferation of all three groups of HDFs was increased by ADSC-Exos (Figure 3(a)). In addition, scratch wound assays were performed to investigate the effect of ADSC-Exos on the migration of HDFs. The stimulative effect on cell migration was determined by evaluating the closure of the scratched area. All three groups showed the same results: the migrating ability of HDFs treated with ADSC-Exos was significantly higher than the control group (Figures 3(b) and 3(c)).

### 3.4. ADSC-Exos Reversed the Expression of ROS and SA-*β*-Gal Activity in HDFs

According to the free radical theory of aging, the leading cause of functional decline is oxidative damage caused by ROS, which is characteristic of aging [32]. After being treated with ADSC-Exos, the expression of ROS was significantly reduced than that of the control (Figure 4(a)).

SA-*β*-Gal is specifically expressed in senescence fibroblast cells, and the expression level of SA-*β*-Gal increases with the senescence in HDFs [33]. It has been the most widely used biomarker for senescent cells because it is reliable and easy to detect. Specific quantitative assays were developed for its detection at pH 6.0. The positive rate of SA-*β*-Gal was inhibited after coculture of senescence HDFs with ADSC-Exos compared to that of the control, as shown in Figures 4(b) and 4(c).

### 3.5. ADSC-Exos Treatment Promoted Type I Collagen Protein Synthesis of HDFs

Type I collagen is the main dermal component, and it is responsible for the tensile strength of the skin tissue. As the skin ages, it gradually loses the contents of type I collagen [34]. In this study, we detected the type I collagen protein level of HDFs. The results showed that type I collagen protein levels of all three groups were increased in the supernatant of HDFs treated with ADSC-Exos compared to those of the untreated HDFs (Figures 5(a) and 5(b)).

### 3.6. ADSC-Exos Inhibited the Expression of Senescence-Related Proteins

In the past years, p16, p21, and p53 have been proved to play important roles in cellular senescence and their protein expression levels were upregulated with cellular senescence [33]. Therefore, the protein expression levels of these three genes were detected by Western blot analyses. Western blot results showed that the protein levels of p16, p21, and p53 had been significantly lower in HDFs treated with ADSC-Exos than in the control group (Figure 6). Moreover, the same results were discovered in the three groups.

## 4. Discussion

The aging of the human skin is a complex process resulting from the interaction between internal mechanisms and external stimuli. Aging is inevitable but can be slightly delayed with the help of science and technology [4]. Due to the burgeoning market demand for antiaging and the growing interest of cosmetic practitioners and plastic surgeons, many treatments have been developed to slow the skin aging process [35]. Adipose-derived stem cells (ADSCs), as one type of mesenchymal stem cells (MSCs), are considered to have antiaging effects and provide a promising and effective option for antiaging facial skin to a certain extent [36]. Compared with other human MSCs, ADSCs are easy to harvest, rapid in culture expansion, and low in immunogenicity, making them an ideal source of extracellular vesicles. Therefore, ADSCs are advantageous for therapeutic applications. However, several issues have hindered the therapeutic use of ADSCs, such as stemness loss and senescence of cells that occur during proliferation [36]. Fortunately, numerous studies have shown that stem cells themselves and their paracrine functional components have potential therapeutic effects on various diseases, in which exosomes play an essential role [37].

Recent studies have shown that exosomes promote wound healing by promoting collagen synthesis and inducing neovascularization in damaged skin [38]. However, the study of ADSC-derived exosomes (ADSC-Exos) on antiaging has been reported rarely. In this study, we have succeeded in isolating exosomes from the ADSC culture medium. We found that by coculturing ADSC-Exos with senescent HDFs in vitro, ADSC-Exos could enhance cellular protein synthesis activity, promote cell migration, and delay cellular senescence.

The expression levels of reactive oxygen species (ROS) and senescence-associated *β*-galactosidase (SA-*β*-Gal) are aging related. Many studies have shown that the most critical factor in cellular senescence is oxidative stress caused by excessive ROS production [31]. Additionally, cellular senescence can also be triggered by high concentrations of ROS [39]. SA-*β*-Gal is a specific biomarker expressed in senescent cells [40]. Human skin biopsies showed that the expression levels of SA-*β*-Gal in dermal fibroblasts and epidermal keratinocytes increased with age [32, 41]. This study found that ADSC-Exos could effectively inhibit excessive ROS and SA-*β*-Gal generation induced by the senescent HDFs during in vitro expansion. These findings suggest that ADSC-Exos can rejuvenate senescent HDFs. Then, we found that ADSC-Exos restored altered expression of collagen type I in senescent HDFs. These results suggest that ADSC-Exos contain beneficial factors that regulate matrix rebalancing in the aging skin and can be successfully delivered to dermal fibroblasts. These factors are thought to regulate the expression of aging-related genes in fibroblasts, enhance the ability of fibroblasts to synthesize type I collagen, increase the content of structural proteins, and promote the reconstruction of the dermal matrix in the aging skin [42].

P16/Rb and p19/p53/p21 are the two most critical signaling pathways in the process of cell senescence [43]. P16, also known as cyclin-dependent kinase inhibitor 2A (CDKN2A), is an important tumor suppressor gene that plays an essential role in cell cycle regulation by inhibiting the G1 phase of cells from entering the S phase [44]. At the same time, with the accumulation of tissue aging and cell division times, the expression of p16 was upregulated [45]. Therefore, p16 is considered an effective biomarker related to cellular senescence and has been applied to detect the degree of human tissue aging at the molecular level. Studies have confirmed that the aging of mice can be delayed by knockout p16 [46]. In addition, p19, p21, and p53 are also essential genes involved in cell senescence [47]. Studies have found that the activity of p53 can be activated when cells undergo senescence and DNA damage and the expression of its protein products gradually increases with the process of cell senescence [48]. P21 is a downstream effector of p53, and the level of p21 protein is also increased in senescent cells [49]. In this study, we demonstrate that the protein expression levels of p53, p21, and p16 were decreased after senescence HDFs treated with ADSC-Exos.

## 5. Conclusions

The human skin undergoes the complex process of aging. Skin aging is unavoidable but can be delayed. ADSCs as potential antiaging agents are being widely studied. However, because of insufficient evidence on safety and efficacy, the use of stem cells in antiaging was limited. Encouragingly, our results have revealed the antisenescence effects of ADSC-Exos on HDFs. Compared with ADSCs, ADSC-Exos have several advantages: being more stably preserved, lower tumorigenicity, and lower immunogenicity. Thus, ADSC-Exos may be a novel cell-free therapeutic tool for antiaging. Of course, more research is needed to demonstrate the therapeutic potential of ADSC-Exos.

## Figures and Tables

**Figure 1:** Identification of ADSCs. (a) Cell morphology of ADSCs. Their cellular morphology tends to be long and stringy. (b) Flow cytometric analysis of cell surface marker expression in ADSCs (CD44, CD73, CD90, CD105, CD34, and CD45). (c) Characterization of isolated ADSCs by adipogenic differentiation. (d) Characterization of isolated ADSCs by osteogenic differentiation. ADSCs: adipose-derived stem cells.

**Figure 2:** Identification of ADSC-Exos. (a) The morphology of exosomes under transmission electron microscopy (TEM). Black bar = 200 nm. Identification of ADSC-Exos. (b) The size distribution and concentration of exosomes were analyzed using nanoparticle tracking analysis (NTA). The mean diameter of ADSC-Exos was 95.16 nm. Identification of ADSC-Exos. (c) Western blotting analysis of exosomal surface marker proteins (including CD9, CD63, and CD81).

**Figure 3:** Proliferation and migration changes of senescence HDFs after being treated with ADSC-Exos. (a) Growth curves of senescence HDFs after being treated with ADSC-Exos. The data shown are expressed as the mean ± SD. ^∗^*P* < 0.05, ^∗∗^*P* < 0.01. Proliferation and migration changes of senescence HDFs after being treated with ADSC-Exos.(b) Cell scratch test of senescence HDFs after being treated with ADSC-Exos (×100). Proliferation and migration changes of senescence HDFs after being treated with ADSC-Exos. (c) Quantitative analysis of the migration area of HDFs. The data shown are expressed as the mean ± SD. ^∗^*P* < 0.05, ^∗∗^*P* < 0.01.

**Figure 4:** ADSC-Exos reversed the expression of ROS and SA-*β*-Gal activity in HDFs. (a) The ROS fluorescence values of the cocultured HDFs. The data shown are expressed as the mean ± SD. ^∗^*P* < 0.05, ^∗∗^*P* < 0.01. ADSC-Exos reversed the expression of ROS and SA-*β*-Gal activity in HDFs. (b) The results of SA-*β*-Gal staining were observed after coculture of HDFs. ADSC-Exos reversed the expression of ROS and SA-*β*-Gal activity in HDFs. (c) Quantitative assays of SA-*β*-Gal staining. The data shown are expressed as the mean ± SD. ^∗^*P* < 0.05, ^∗∗^*P* < 0.01.

**Figure 5:** ADSC-Exos treatment promoted type I collagen protein synthesis of HDFs. (a) The standard curve of human type I collagen. ADSC-Exos treatment promoted type I collagen protein synthesis of HDFs. (b) Using the ELISA kit to analyze the content of type I collagen. The data shown are expressed as the mean ± SD. ^∗^*P* < 0.05, ^∗∗^*P* < 0.01.

**Figure 6:** ADSC-Exos inhibited the expression of senescence-related proteins. Western blot detected the expression of senescence-associated proteins (p16, p21, and p53) in fibroblasts. ADSCs: adipose-derived stem cells; ADSC-Exos: ADSC-derived exosomes.

## Data Availability

Some or all data, models, or code generated or used during the study are available from the corresponding author by request.

## References

[1] Zhang S., Duan E. (2018). Fighting against skin aging: the way from bench to bedside. *Cell Transplantation*.

[2] Haydont V., Bernard B. A., Fortunel N. O. (2019). Age-related evolutions of the dermis: clinical signs, fibroblast and extracellular matrix dynamics. *Mechanisms of Ageing and Development*.

[3] Maisel-Campbell A. L., Ismail A., Reynolds K. A. (2020). A systematic review of the safety and effectiveness of platelet-rich plasma (PRP) for skin aging. *Archives of Dermatological Research*.

[4] Kohl E., Steinbauer J., Landthaler M., Szeimies R. M. (2011). Skin ageing. *Journal of the European Academy of Dermatology and Venereology*.

[5] Rippa A. L., Kalabusheva E. P., Vorotelyak E. A. (2019). Regeneration of dermis: scarring and cells involved. *Cells-Basel*.

[6] Kazanci A., Kurus M., Atasever A. (2017). Analyses of changes on skin by aging. *Skin Research and Technology*.

[7] Shin J. W., Kwon S. H., Choi J. Y. (2019). Molecular mechanisms of dermal aging and antiaging approaches. *International Journal of Molecular Sciences*.

[8] Pu X., Ma S., Gao Y., Xu T., Chang P., Dong L. (2021). Mesenchymal Stem Cell-Derived Exosomes: Biological Function and Their Therapeutic Potential in Radiation Damage. *Cells-Basel*.

[9] Levy O., Kuai R., Siren E. (2020). Shattering barriers toward clinically meaningful MSC therapies. *Science Advances*.

[10] Al-Khawaga S., Abdelalim E. M. (2020). Potential application of mesenchymal stem cells and their exosomes in lung injury: an emerging therapeutic option for COVID-19 patients. *Stem Cell Research & Therapy*.

[11] Yu K., Zeng Z., Cheng S. (2020). TPP1 enhances the therapeutic effects of transplanted aged mesenchymal stem cells in infarcted hearts via the MRE11/AKT pathway. *Frontiers in Cell and Development Biology*.

[12] Keshtkar S., Azarpira N., Ghahremani M. H. (2018). Mesenchymal stem cell-derived extracellular vesicles: novel frontiers in regenerative medicine. *Stem Cell Research & Therapy*.

[13] Mendt M., Rezvani K., Shpall E. (2019). Mesenchymal stem cell-derived exosomes for clinical use. *Bone Marrow Transplantation*.

[14] Zouboulis C. C., Makrantonaki E., Nikolakis G. (2019). When the skin is in the center of interest: an aging issue. *Clinics in Dermatology*.

[15] Bjorge I. M., Kim S. Y., Mano J. F., Kalionis B., Chrzanowski W. (2017). Extracellular vesicles, exosomes and shedding vesicles in regenerative medicine - a new paradigm for tissue repair. *Biomaterials Science*.

[16] Zhao B., Li X., Shi X. (2018). Exosomal micro RNAs derived from human amniotic epithelial cells accelerate wound healing by promoting the proliferation and migration of fibroblasts. *Stem Cells International*.

[17] Tran P., Xiang D., Tran T. (2020). Exosomes and nanoengineering: a match made for precision therapeutics. *Advanced Materials*.

[18] Pegtel D. M., Gould S. J. (2019). Exosomes. *Annual Review of Biochemistry*.

[19] Zhuang L., Xia W., Chen D. (2020). Exosomal LncRNA-NEAT1 derived from MIF-treated mesenchymal stem cells protected against doxorubicin-induced cardiac senescence through sponging miR-221-3p. *J Nanobiotechnology*.

[20] Xiao W., Tang H., Wu M. (2017). Ozone oil promotes wound healing by increasing the migration of fibroblasts via PI3K/Akt/mTOR signaling pathway. *Bioscience Reports*.

[21] Casado-Diaz A., Quesada-Gomez J. M., Dorado G. (2020). Extracellular vesicles derived from mesenchymal stem cells (MSC) in regenerative medicine: applications in skin wound healing. *Frontiers in Bioengineering and Biotechnology*.

[22] Giassafaki L. N., Siqueira S., Panteris E. (2021). Towards analyzing the potential of exosomes to deliver microRNA therapeutics. *Journal of Cellular Physiology*.

[23] Xu R., Greening D. W., Zhu H. J., Takahashi N., Simpson R. J. (2016). Extracellular vesicle isolation and characterization: toward clinical application. *The Journal of Clinical Investigation*.

[24] Hoang D. H., Nguyen T. D., Nguyen H. P. (2020). Differential wound healing capacity of mesenchymal stem cell-derived exosomes originated from bone marrow, adipose tissue and umbilical cord under serum- and xeno-free condition. *Frontiers in Molecular Biosciences*.

[25] Wu D., Kang L., Tian J. (2020). Exosomes derived from bone mesenchymal stem cells with the stimulation of Fe nanoparticles and static magnetic field enhance wound healing through upregulated miR-21-5p. *International Journal of Nanomedicine*.

[26] Yaghoubi Y., Movassaghpour A., Zamani M., Talebi M., Mehdizadeh A., Yousefi M. (2019). Human umbilical cord mesenchymal stem cells derived-exosomes in diseases treatment. *Life Sciences*.

[27] Stahl P. D., Raposo G. (2019). Extracellular vesicles: exosomes and microvesicles, integrators of homeostasis. *Physiology (Bethesda)*.

[28] Ratajczak M. Z., Ratajczak J. (2020). Extracellular microvesicles/exosomes: discovery, disbelief, acceptance, and the future?. *Leukemia*.

[29] O’Brien K., Breyne K., Ughetto S., Laurent L. C., Breakefield X. O. (2020). RNA delivery by extracellular vesicles in mammalian cells and its applications. *Nature Reviews. Molecular Cell Biology*.

[30] Thery C., Amigorena S., Raposo G., Clayton A. (2006). Isolation and characterization of exosomes from cell culture supernatants and biological fluids. *Current Protocols In Cell Biology*.

[31] Liao N., Shi Y., Zhang C. (2019). Antioxidants inhibit cell senescence and preserve stemness of adipose tissue-derived stem cells by reducing ROS generation during long-term in vitro expansion. *Stem Cell Research & Therapy*.

[32] Sasaki M., Kajiya H., Ozeki S., Okabe K., Ikebe T. (2014). Reactive oxygen species promotes cellular senescence in normal human epidermal keratinocytes through epigenetic regulation of p16^INK4a^. *Biochemical and Biophysical Research Communications*.

[33] Noren H. N., Evans M. K. (2017). Techniques to induce and quantify cellular senescence. *Journal of Visualized Experiments*.

[34] Purohit T., He T., Qin Z. (2016). Smad3-dependent regulation of type I collagen in human dermal fibroblasts: impact on human skin connective tissue aging. *Journal of Dermatological Science*.

[35] Liu T., Li N., Yan Y. Q. (2020). Recent advances in the anti-aging effects of phytoestrogens on collagen, water content, and oxidative stress. *Phytotherapy Research*.

[36] Zarei F., Abbaszadeh A. (2019). Application of cell therapy for anti-aging facial skin. *Current Stem Cell Research & Therapy*.

[37] Ha D. H., Kim H. K., Lee J. (2020). Mesenchymal Stem/Stromal Cell-Derived Exosomes for Immunomodulatory Therapeutics and Skin Regeneration. *Cells-Basel*.

[38] Laberge A., Arif S., Moulin V. J. (2018). Microvesicles: intercellular messengers in cutaneous wound healing. *Journal of Cellular Physiology*.

[39] Ruan Y., Jiang S., Gericke A. (2021). Age-related macular degeneration: role of oxidative stress and blood vessels. *International Journal of Molecular Sciences*.

[40] Zhang Y., Xu J., Liu S. (2019). Embryonic stem cell-derived extracellular vesicles enhance the therapeutic effect of mesenchymal stem cells. *Theranostics*.

[41] Kim J. Y., Lee S. H., Ahn Y. (2020). Role of senescent fibroblasts in the development of idiopathic guttate hypomelanosis. *The British Journal of Dermatology*.

[42] Eylert G., Dolp R., Parousis A. (2021). Skin regeneration is accelerated by a lower dose of multipotent mesenchymal stromal/stem cells-a paradigm change. *Stem Cell Research & Therapy*.

[43] Zhang W., Yang J., Chen Y. (2021). Lycorine hydrochloride suppresses stress-induced premature cellular senescence by stabilizing the genome of human cells. *Aging Cell*.

[44] He S., Sharpless N. E. (2017). Senescence in health and disease. *Cell*.

[45] LaPak K. M., Burd C. E. (2014). The molecular balancing act of p16 (INK4a) in cancer and aging. *Molecular Cancer Research*.

[46] Yousefzadeh M. J., Zhao J., Bukata C. (2020). Tissue specificity of senescent cell accumulation during physiologic and accelerated aging of mice. *Aging Cell*.

[47] Jiang C., Liu G., Luckhardt T. (2017). Serpine 1 induces alveolar type II cell senescence through activating p53-p21-Rb pathway in fibrotic lung disease. *Aging Cell*.

[48] Kon N., Ou Y., Wang S. J., Li H., Rustgi A. K., Gu W. (2021). Corrigendum: mTOR inhibition acts as an unexpected checkpoint in p53-mediated tumor suppression. *Genes & Development*.

[49] Xu S., Wu W., Huang H. (2019). The p53/miRNAs/Ccna2 pathway serves as a novel regulator of cellular senescence: complement of the canonical p53/p21 pathway. *Aging Cell*.

